# The Ottawa Decision-Making Supportive Framework-Based Nursing Care in the Outcome of Patients with Chronic Heart Failure

**DOI:** 10.1155/2022/6000160

**Published:** 2022-09-26

**Authors:** Yufang Teng, Tingting Liu, Xiaxia Li, Weilu Feng, Yanping Wu, Shan Su, Xiaobo Guan

**Affiliations:** ^1^Department of Cardiovascular Medicine, Lanzhou First People's Hospital, Lanzhou 730050, Gansu, China; ^2^CT Room, Lanzhou First People's Hospital, Lanzhou 730050, Gansu, China

## Abstract

**Objective:**

To examine the psychological, compliance, and prognostic impact of care based on the Ottawa Decision Support Framework on patients with chronic heart failure.

**Methods:**

The medical profiles of 80 individuals with permanent heart failure from January 2020 to January 2021 were retrospectively analyzed. The care was provided in the framework of Ottawa Decision Support alongside the clinical standard of care. The self-assessment anxiety scale (SAS), Frankel treatment adherence scale, Minnesota quality of life questionnaire for heart failure, self-care competence scale (ESCA), complication rates, and readmission rates were compared prior to and postcare.

**Results:**

Following three-month nursing care, the score of the SAS scale was remarkably fewer, and the difference was statistically significant (*P* < 0.05). Three months of care later, the scores on the Frank Scale were substantially superior to those before care, and the difference was statistically significant (*P* < 0.05). Aftercare, the Minnesota quality of life questionnaire for heart failure was clearly inferior to precare, and the difference was statistically significant (*P* < 0.05). The ESCA scale scores were found to be considerably more favorable after three months of care than before care, and the difference was statistically significant (*P* < 0.05). After nursing care, one arrhythmia (1.25%) and one pulmonary infection (1.25%) were noted, and the difference was statistically significant (*P* < 0.05). The prevalence of complications was 2.50%, and the difference was statistically significant (*P* < 0.05). Three cases were readmitted for recurrent chronic heart failure, which was a 2.75% readmission rate.

**Conclusion:**

Continuous nursing based on the Ottawa Decision Support Framework has significant application value in an anxiety state, treatment compliance, and prognosis of patients with chronic heart failure, which can more effectively reduce patients' anxiety and the incidence of complications and readmission rate, in the meanwhile, effectively improve treatment compliance, quality of life, self-care ability, and prognosis, which is worthy of clinical application.

## 1. Introduction 

Chronic heart failure is part of the end stage of various cardiac diseases. The abnormalities in the structure and function of the heart caused by different types of heart disease affect ventricular filling and ejection function, reduce cardiac output and lead to an increase in pulmonary venous pressure. There are varying degrees of deterioration and premature death of cardiomyocytes [1, 2]. It has become one of the most important medical and public health issues today and it is imperative to prevent and treat heart failure. In recent years, great progress has been made in the pharmacological and surgical treatment of heart failure, but the symptoms of dyspnea, fatigue, and edema in patients with heart failure have not been well controlled. Although patients receive medical interventions during their stay in the hospital, they have a role to play in improving their quality of life [3]. The statistics have shown that the number of patients with cardiovascular disease (CVD) in the Chinese population is about 290 million, including about 4.5 million patients with chronic heart failure. The mortality rate of CVD is the leading cause of death in China, accounting for about 40% [4]. With the aging of the population in China, chronic heart failure has become one of the diseases that seriously threaten the health of our people [5].

At present, there is no unified treatment plan for the treatment of chronic heart failure and the main treatment is to alleviate clinical symptoms and control the progress of the disease [6]. For patients with chronic diseases, establishing a long-term doctor-patient relationship can improve communication, deepen the understanding of the patient's medical history by care providers, and thereby effectively manage chronic diseases and establish long-term disease monitoring mechanisms [7]. A few studies have shown that the clinical treatment of patients with chronic heart failure is a long process and has an increase in recurrence rate [8, 9]. Therefore, the healthcare needs of patients with chronic heart failure after discharge are still relatively high. However, the current community nursing system in China is not perfect. Patients with chronic heart failure usually do not get effective nursing support after discharge. Only when the disease develops to a certain extent can they seek medical treatment.

In the late 1990s, researchers such as Naylor et al. thought that the condition of patients should be evaluated after they were discharged from the hospital, not only for mental intervention but also for patients' families to learn some nursing knowledge and health knowledge [10, 11]. The results showed that by giving this nursing method, the probability of readmission could be significantly reduced and the quality of life of patients could be significantly improved. At the beginning of the 21st century, researcher Freeman et al. put forward a model after in-depth research, which included six dimensions [12]. After in-depth research, Hagger-ty et al. published that continuous nursing was expounded and its two core elements were analyzed. One was the continuation of nursing service time, the other was the continuation of health service [13].

In 1989, Professor Annette O'Connor of the University of Ottawa wrote in his book Nursing diagnosis and intervention that patients sometimes raise decision-making needs, such as being skeptical about the effectiveness of treatment and exploring how to deal with the situation [14]. The Ottawa Decision Support Framework research work was funded by the Canadian Institutes of Health and the Canadian lead researcher program [15]. The research included investigating decision-making needs, designing and evaluating decision support tools/methods such as decision assistance tools and decision guidance and developing and evaluating training programs to improve clinicians' ability to implement decision support. It can decompose the complex evidence application process into several specific and enforceable stages, which can provide direction for problem solving and action planning, and achieve remarkable results in clinical application [16]. A continuous nursing model can provide continuous nursing and health-related knowledge for chronic heart failure after discharge and meet the nursing needs of chronic heart failure after discharge. The continuous nursing model based on the Ottawa Decision Support Framework is a new nursing model that applies Ottawa Decision Support Framework to continuous nursing service. It can guide clinical nurses to carry out continuous nursing work for patients with chronic heart failure. Therefore, the clinical data of 80 patients with chronic heart failure from January 2020 to January 2021 were analyzed retrospectively to study the value of continuous nursing based on the Ottawa Decision Support Framework in improving anxiety, treatment compliance, and prognosis.

## 2. Materials and Methods

### 2.1. General Information

The clinical data of 80 patients with chronic heart failure from January 2020 to January 2021 were analyzed. 80 patients with chronic heart failure received continuous nursing based on the Ottawa Decision Support Framework on the basis of clinical systematic treatment. Among the 80 patients, there were 40 males and 40 females, whose ages ranged from 58 to 77 years old with a mean age of 61.12 ± 5.23.

#### 2.1.1. Inclusion Criteria

Inclusion criteria were as follows: (1) patients with chronic heart failure diagnosed in accordance with the guidelines for diagnosis and treatment of Heart failure in 2018; (2) AHA cardiac function grade II-III; (3) activities of daily living (ADL) score < 22; (4) patients who could be discharged; (5) age ≥ 60 years old with primary school education or above; (6) patients living in this city.

#### 2.1.2. Exclusion Criteria

Exclusion criteria were as follows: (1) patients with chronic heart failure, in the end, stage complicated with malignant diseases; (2) patients with chronic heart failure complicated with other serious diseases of the system; (3) patients with obvious limb dysfunction; (4) patients with cognitive impairment (SPMSQ).

#### 2.1.3. Termination Criteria

Patients who were unwilling to continue to cooperate during the study or who had accidents/died from various causes.

### 2.2. Methods

#### 2.2.1. Technical Route

As shown in Figure 1.

#### 2.2.2. Treatment Methods

After admission, 80 patients with chronic heart failure received symptomatic treatment, such as reducing blood pressure, antiplatelet aggregation, correcting acid-base and water-electrolyte imbalance, reducing blood pressure, regulating lipids, and so on.

#### 2.2.3. Nursing Methods

All 80 patients received basic care, such as ensuring the ward environment, regular disinfection and ventilation, 24-hour ambulatory ECG monitoring, recording patients' vital signs, and notifying doctors immediately if abnormalities were detected. Prepare for first aid and handle emergencies appropriately. Active prevention of complications such as infection, turning and patting the back every 2 hours, and keeping the skin clean and dry.

On this basis, continuous nursing based on the framework of Ottawa decision support was implemented. (1) Explore nursing demonstration: set up a continuous nursing group based on the Ottawa Decision Support Framework. The decision guidance, the International Cooperative Organization for patient decision assistance tools, and its standard development were based on the continuous nursing manual under the Ottawa Decision Support Framework. (2) Clarify decision assessment/discussion decision needs: the patients were ensured to accurately understand decision-making problems, and evaluate the decision-making stage. (3) Decision-making nursing plan: Ottawa studies the application of continuous nursing measures of the application model. Before nursing implementation, the members of the group were ensured to understand the content and function of the continuous nursing plan and have the ability to promote the transformation of the continuous nursing plan into practice. During the nursing implementation, the researchers needed to continuously evaluate the willingness of the members of the group to practice to promote the smooth implementation of the continuous nursing plan. To assess patient understanding and assess facts: options, benefits, hazards/risks/side effects, probabilities. Identify values, assess the value/importance of different outcomes, clarify values, promote communication about values, use scales with scores ranging from 0 (very unimportant) to 5 (very important), and ask patients about their preferences. (4) Make clear the decision-making needs. Assess/discuss decision-making needs and evaluate the role of others in decision-making (views, support, and stress). Building skills and confidence in implementing decision-making steps, communicating preferences and dealing with stress, and using affirmative scale entries to assess decision-making needs. (5) Plan the next steps based on the requirements. Promote the decision-making process, promote plan-making, and deal with the decision-making needs to be solved. Identify the conditions required to implement this preference, talk to patients about their views on sharing personal preferences with healthcare staff, and develop skills for deliberation, communication, and support. One day before discharge, the research team evaluated the patients comprehensively according to the decision guidance based on Ottawa personal decision guidelines, focusing on the possible nursing problems and corresponding nursing measures after discharge. Patients were evaluated and intervened with a continuous care program based on the Ottawa Decision Support Framework during telephone follow-up and home follow-up. If patients had nursing problems, family visits could be conducted at any time for on-site one-to-one guidance.

### 2.3. Observation Index

The main results were as follows:

1. The scores of the self-rating anxiety scale (SAS) before and 3 months after nursing were analyzed. There were 20 items on the SAS scale [17], including 15 positive score items and 5 reverse score items. The standard score ≥ 50 was regarded as anxiety, 50 ≤ SAS < 60 as mild to mild anxiety, 60 ≤ SAS < 70 as moderate anxiety, and SAS ≥ 70 as severe anxiety. With the increase in the score, the degree of anxiety is more serious.
2. The scores of the Frankl treatment compliance scale before nursing and 3 months after nursing were analyzed. The score criteria of the Frankl compliance scale [18] were as follows: 1: refusal, pain; 2: uncooperation and reluctance; 3: use, indifference; 4: active cooperation and enjoyment. The higher the score, the better compliance.
3. The scores of the Minnesota heart failure quality of life questionnaire before nursing and 3 months after nursing were analyzed. The physical limitation, emotion, clinical symptoms, and social limitations of the patients were evaluated according to the Minnesota chronic heart failure quality of life questionnaire [2]. Each item indicated the effect of heart failure on the patient's life quality. The score was from 0 to 5 and the total score was 0–20.
4. The scores of the self-nursing ability scale (ESCA) before nursing and 3 months after nursing were analyzed. The ESCA scale [19] included 4 evaluation items and 43 items, including self-concept (8 items), sense of self-care responsibility (6 items), self-nursing skills (12 items), and health knowledge level (17 items). The scale was scored with a scale of 0–4 points and 5 grades, including 4 points: very much like me; 3 points: a little like me; 2 points: uncertain; 1 point: some are not like me; 0 points: very unlike me. The total score is 172.
5. To analyze the incidence of complications and the rate of readmission after 3 months of nursing.

### 2.4. Statistical Analysis

IBMSPSS24.0 software was applied for statistical analysis. The measurement data were expressed by mean ± standard deviation. The counting data were expressed by frequency or rate. *T*-test was used when measurement data obey normal distribution, and rank sum test was used when it did not obey normal distribution. *χ*^2^ test was used to compare the classified counting data. Repeated measurement data were analyzed by repeated measurement analysis of variance. Main effect test results were used when there was no interaction and simple effect analysis was carried out when there was interaction. *P* < 0.05 indicated that the difference between groups is statistically significant.

## 3. Results

### 3.1. Analysis of SAS Scale Score before Nursing and 3 Months after Nursing

After nursing for 3 months, the score of SAS was significantly lower than that before nursing, and the difference was statistically significant (*P* < 0.05). See Table 1.

### 3.2. Analysis of Frank Scale Score before Nursing and 3 Months after Nursing

After 3-month nursing care, the score of the Frank scale was significantly higher than that before nursing, and the difference was statistically significant (*P* < 0.05). See Table 2.

### 3.3. Analysis of the Life-Quality Questionnaire Score of Minnesota Heart Failure before Nursing and 3-Month Nursing Care

After 3-month nursing care, the score of the Minnesota heart failure quality of life questionnaire was significantly lower than that before nursing, and the difference was statistically significant (*P* < 0.05). See Table 3.

### 3.4. Analysis of ESCA Scale Score before Nursing and 3 Months after Nursing

After 3-month nursing care, the score of the ESCA scale was significantly higher than that before nursing, and the difference was statistically significant (*P* < 0.05). See Table 4.

### 3.5. To Analyze the Incidence of Complications and the Rate of Readmission after 3-Month Nursing Care

After 3 months of nursing in 80 patients, one case (1.25%) developed an arrhythmia, one case (1.25%) had a pulmonary infection and the complication rate was 2.50%. The admission rate was 2.75%. See Table 5.

## 4. Discussion

Clinical studies have shown that chronic heart failure is a severe and terminal stage of various cardiovascular diseases characterized by high prevalence, high mortality, and high readmission rate [20–23]. The physical and mental health of patients can reduce their quality of life and the medical expenses caused by repeated hospitalization have brought a heavy economic burden to the family and society [24]. The patients mainly showed decreased exercise endurance (fatigue and dyspnea), body fluid retention (pulmonary congestion and limb edema), and so on. The epidemiology of chronic heart failure has shown that the incidence and mortality of chronic heart failure are positively correlated with age, especially in patients ≥ 70 years old. The incidence is as high as 30.8% [25]. However, after the acute phase in patients with chronic heart failure, the cardiac rehabilitation period is longer. Therefore, it is clear that the community, family, and medical care are all within the scope of the rehabilitation environment. After discharge, if the patient is unable to care for themselves, this will affect their condition increasing the risk of readmission [26–28]. This paper was to study the value of continuous nursing based on the Ottawa Decision Support Framework in improving anxiety, treatment compliance, and prognosis.

Ongoing care research has been undertaken in many of our hospitals to address this issue. Chronic conditions, if not managed effectively, can lead to acute exacerbations of chronic conditions and associated complications, increasing patient readmission rates. Continuing care can prevent short-term hospitalization of older people with chronic conditions [29]. According to the traditional view, the care of patients with chronic heart failure is limited to their hospitalization and they will stop providing nursing services after discharge, however, many patients with chronic heart failure still have a variety of health problems at discharge [30]. By giving them continuous nursing care, patients can also receive professional nursing intervention outside the hospital, so as to improve the recovery effect, and scientifically objectively assessing the needs of patients with chronic heart failure is an important part of establishing a complete continuous nursing system. At present, the continuum of care has been explored for over 20 years and has resulted in a series of specific theories and guidance models [31, 32]. At present, the methods of extended care mainly include discharge guidance, home visits, telephone follow-up, and the establishment of extended care centers [33, 34]. However, each type of continuous care has its own advantages and limitations [35]. With the development of modern evidence-based medicine, an evidence-based theoretical framework for guiding patients to make clinical decisions—the Ottawa Decision Support Framework came into being. The Ottawa Theory aims to provide an interdisciplinary and comprehensive research framework applicable to any level of organization, medical service, and healthcare system to help researchers conduct scientific research [36]. Therefore, this article conducted a study to investigate the anxiety status, treatment adherence, and prognostic value of the continuum of care under the Ottawa Decision Support Framework for chronic heart failure patients.

Continuous nursing is a way to provide patients with a series of measures to provide patients with different levels of care so that patients can get continuous care. Under normal circumstances, it refers to patients receiving care at home, such as community follow-up of patients, and guidance for discharged patients. The results showed that after implementing continuous care based on the Ottawa decision support framework, the patients' SAS scale scores were significantly lower than those before care (*P* < 0.05). The Frank scale score was significantly higher than that before nursing, and the difference was statistically significant (*P* < 0.05). Minnesota heart failure quality of life questionnaire scores were significantly lower than those before nursing (*P* < 0.05). The ESCA scale score of the patients was significantly higher than that before nursing, and the difference was statistically significant (*P* < 0.05). After 3-month nursing care, there was 1 case of arrhythmia (1.25%) and 1 case of pulmonary infection (1.25%). The incidence of complications was 2.50%. 3 cases were readmitted to the hospital because of recurrence of chronic heart failure and the readmission rate was 2.75%. The patient's anxiety is reduced and treatment compliance is enhanced. Patients' quality of life is improved and as a result, complication rates and readmission rates are reduced. The Ottawa Decision Support Framework is an evidence-based, practical, and neutral theory to guide patients in making health or social decisions [37]. Through the establishment of a continuous nursing team based on the Ottawa Decision Support Framework. The Ottawa Decision Support Framework-based continuum of care has proven to be of significant value in the application of anxiety states, treatment adherence, and prognosis in patients with chronic heart failure.

Based on the literature review and the Ottawa Decision Support Framework, the IOM's patient decision aid tool and its standards are based on the Continuum of Care manual under the Ottawa Decision Support Framework. Patients are helped to acquire the skills to participate in decision-making, including considering various treatment options and discussing with their doctors the implementation of selected decision-making options to meet their needs for self-management knowledge. Patients are given more scientific guidance on self-management behaviors. Patients are invited to actively participate in the scientific adaptation and modification of care programs, taking into account their opinions and suggestions. These measures can reduce or eliminate decision-making conflicts and address patients' poor cognitive abilities, poor compliance, and high anxiety. In addition, in the process of building the system, this study invited patients to participate actively, evaluated the needs and obstacles of patients, and embodies the service concept of “patient-centered,” as well as medical humanistic care. In addition, patients are in an active position in nursing, which can promote patients to actively participate in treatment decisions, significantly enhance patients' enthusiasm for learning and improve patients' ability and compliance with self-maintenance behavior in health management, so as to reduce the occurrence of complications [38, 39]. There are some limitations to this study. First, the sample size of this study is not large and it is a single-center study, so bias is inevitable. In future research, we will carry out multicenter, large-sample prospective studies, or more valuable conclusions can be drawn.

To sum up, continuous nursing care which is based on the Ottawa Decision Support Framework has valuable applications in the anxiety status, therapeutic compliance, and survival of patients with chronic heart failure. It is recommended for further use in clinical settings as it is capable of reducing patient anxiety, reducing complications, and readmission rates, while effectively enhancing therapeutic compliance and prognosis.

## Figures and Tables

**Figure 1:** Technology roadmap.

**Table 1:** Analysis of prenursing and 3-month nursing SAS scale scores (*n* = 80).

Time	SAS scale score (points)
Before nursing	58.38 ± 5.47
Nursing for 3 months	41.65 ± 3.11
*t* Value	23.781
*P* value	*P* < 0.05

**Table 2:** Frank score of prenursing and 3-month nursing care (*n* = 80).

Time	Frank scale score (points)
Before nursing	2.44 ± 0.18
Nursing for 3 months	3.71 ± 0.06
*t* Value	3.646
*P* value	*P* < 0.05

**Table 3:** Analysis of the life-quality questionnaire score of Minnesota heart failure before nursing and 3 months after nursing (*n* = 80).

Time	Minnesota heart failure quality of life questionnaire score (points)
Before nursing	16.38 ± 3.26
Nursing for 3 months	10.45 ± 1.18
*t* Value	15.298
*P* value	*P* < 0.05

**Table 4:** ESCA score of prenursing and 3-month nursing (*n* = 80).

Time	ESCA scale score (points)
Before nursing	65.54 ± 4.13
Nursing for 3 months	101.85 ± 8.89
*t* Value	33.131
*P* value	*P* < 0.05

**Table 5:** Analysis of complication rate and readmission rate after 3 months of nursing (*n* = 80).

Type of complication	Patients with complications (cases/)	Complication rate (cases/%)	Readmission rate (cases/%)
Arrhythmia	1/1.25	2/2.50	3/2.75
Lung infection	1/1.25		
Thromboembolism	0/0.00		

## Data Availability

The datasets used and analyzed during the current study are available from the corresponding author upon reasonable request.
